# Exploring the Employment Quality Evaluation Model of Application-Oriented University Graduates by Deep Learning

This article has been retracted.

**DOI:** 10.1155/2022/2823614

**Published:** 2022-04-23

**Authors:** Yiran He, Wanhong Zhang, Weiming Xu, Xinru Sui

**Affiliations:** ^1^School of Public Policy & Management, School of Emergency Management, China University of Mining and Technology, Xuzhou 221000, China; ^2^Ludong University, Yantai, Shandong 264000, China; ^3^Yantai Natural Museum, Yantai, Shandong 264000, China

## Abstract

In view of the employment difficulties of college graduates, this paper analyzes the overflow of graduates in a particular period caused by the expansion of enrollment in various colleges and universities and the social phenomenon of social positions in short supply. First, the employment status of application-oriented college students and the deficiencies of employment guidance courses are summarized. Then, deep learning technology is combined with the relevant employment concept to construct an employment training model to guide college students in employment. Besides, a questionnaire on learning effect and employment quality is designed from four perspectives: learning motivation, concentration, teaching process, and final results. The information collected through the questionnaire demonstrates that the employment quality and learning effect of male and female students are not significantly affected by gender differences. In addition, the *P* values of learning motivation, concentration, and teaching process are all less than 0.01, and the unstandardized coefficient of the teaching process is 0.349, which has the most significant impact on the learning effect. In short, the three factors positively affect the learning effect. Therefore, it comes to the conclusion of improving the ability and strategy of classroom employment guidance. If one wants to be successful in job hunting and career selection, it is not enough just to be competitive but also to be good at it. Being good at the competition is reflected in having good psychological quality, strength, and a good competitive state. In the job hunting and career selection competition, attention should be paid to whether the expected value is appropriate. College students should have sufficient self-awareness before preparing to submit resumes. During the interview, they should overcome emotional anxiety. If a person can treat study, work, and life in a good mood from beginning to end, he will win the competition. The research reported here can provide some reference suggestions for the employment quality of application-oriented college graduates.

## 1. Introduction

In the ten years since the implementation of the education reform policy in China, many domestic higher education institutions have begun to change from elite education for individuals to all-around education for the public. Many postsecondary specialized colleges have been promoted to undergraduate colleges and universities and developed rapidly. Moreover, colleges and universities have begun to pay attention to cultivating students' comprehensive quality [1]. However, with the increasing number of college students admitted year by year, the employment situation of graduates in the same period has become even grimmer. Although the government and relevant departments have issued a series of policies to promote graduates' employment in time, it is still challenging to solve difficult employment and uneven employment quality [2]. Therefore, specific educational institutions need to cultivate their educational strategies to improve the employment quality of graduates, which has become a hot research topic.

With the expansion of college enrollment, meritocratic education is gradually spreading to the masses. Niu et al. (2020) believed that the experience of higher education and elite education could break or strengthen the connection between social origin and status acquisition in elite society. Besides, elite management could play a role in the trajectories of graduate study and employment [3]. This research shows that elite education can help students obtain better employment opportunities, and application-oriented universities exemplify the rationality of elite education. Li and Xue (2021) agreed that introducing international academic peer review and tenure tracking mechanisms into China's current higher education system was necessary to achieve the international educational standards pursued by world-class universities, especially in a fiercely global competitive environment [4]. Singh and Miah (2019) thought that research on mobile applications in education by technologies such as mobile learning was still in its infancy, and formal methods for deep learning management systems to support students and scholars to meet industry needs were still to be developed by higher education institutions [5]. Lv et al. (2020) made an effort to find a cognitive computing technology to effectively learn and process large-scale data considering massive data generated with the continuous expansion of data scale [6]. Lv et al. (2020) adopted an improved general spatial pattern algorithm combined with transfer learning, reflecting a good classification effect in both public spatial patterns, indicating that the deep learning algorithm could provide new ideas for innovative teaching [7]. Ran and Xu (2019) found that teachers' teaching characteristics had different effects on college students' grades and future employment quality [8]. The authors found the influencing factors of college students' employment quality from a third-party perspective. Scott et al. (2019) recognized the importance of graduates having appropriate employability skills and subject-specific skills. Therefore, the authors adopted a specific employability skills development strategy for honor students. The module has been perceived to be highly useful, resulting in significant increases in students' confidence across key areas of employability skills [9]. Hernández-Sánchez et al. (2020) found that, during the COVID-19 pandemic, surrounding external factors had a disproportionately destructive impact on the mental health of college students, and the enthusiasm and optimism of college students themselves had a significant effect on employment intentions [10]. Through the above literature research, it can be found that there are many factors affecting the elite education and applied education of college students and ultimately leading to uneven employment quality.

This paper analyzes the factors influencing the employment quality of application-oriented college students. First, the status quo of the employment quality of college graduates is analyzed. There is a prominent contradiction between the rapid increase in the number of graduates and the supply and demand structure with limited short-term growth in social effective demand. Affected by the long-term planned economy and elite education, some graduates have deviations in their career choices. There is a big gap between their employment expectations and social needs. The basic awareness and entrepreneurial awareness of graduates need to be strengthened. Detailed and in-depth ideological education and employment guidance are urgently needed. Then, the feasibility of applying deep learning technology to the college graduates' employment training is discussed. Moreover, an employment training strategy model of college graduates is constructed based on the effectiveness of the deep learning technology. A questionnaire for employment guidance for graduates is designed through the employment impact measurement and other theoretical knowledge. This questionnaire verifies the performance of the employment guidance model. The research innovation lies in combining deep learning with questionnaires to explore the subjective attitudes of students and put forward specific improvement suggestions. The employment of graduates is related to the interests of millions of people and the stability and harmony of society. The current economic development must be carefully analyzed from the perspective of learning and practicing the scientific concept of development. Therefore, the pertinence and effectiveness of the policy will be improved. The conclusion is that the reasonable planning of graduates' careers is the first step for college students to succeed, which is of great significance. It guides graduates to correctly understand their personality traits and accurately locate their value. It enables graduates to clarify their ideal career and development goals and find a suitable career path. In addition, it guides graduates to explore their potential advantages and enhance their employment competitiveness. Also, it enables them to face the constantly changing society and enhance their adaptability.

## 2. Methods

### 2.1. Employment Status of University Graduates

With the issuance of the policy of expanding enrollment in colleges and universities in China, the low registration rate of first-year students for several consecutive years has made junior colleges feel the colossal pressure of “not to advance is to die.” Hence, these schools have adopted all means to promote undergraduate colleges to enjoy the dividend of large-scale enrollment expansion. After a leap in enrollment expansion, the annual enrollment scale is still rising so that all colleges and universities taste the benefits of upgrading. However, colleges and universities almost ignore the continuously declining employment rate and quality of employment because of the crowded enrollment situation. Therefore, the number of college graduates each year is much higher than the number required by various positions in society. As a result, many college students are unable to find employment. Meanwhile, job spillovers lead to unemployment [11], finally leading to the vicious circle of employment as shown in Figure 1.

Enterprises follow the laws of the market. Job seekers cannot blame employers. However, the school regards the internship as a teaching link and calculates the credits. Then, they should help employed college students find internship units and give guidance at any time during the internship process. However, the employment of college students looking for internships is entirely on their own, and the school provides only a letter of introduction. During the internship period, the school seldom pays attention to the employment situation of students. Many vocational colleges now have student internship bases. For undergraduates in comprehensive universities, internship and employment are quite difficult issues. Therefore, all colleges and universities must realize the harm of this blind enrollment expansion and break this vicious circle in time.

As the last instructor of graduates, teachers need to guide graduates to a certain degree in the concept of employment. Therefore, whether teachers have received the correct employment guidance courses for graduates will also affect the employment quality of graduates to a certain extent [12]. However, according to the survey, not many teachers have received training in career guidance courses in domestic universities.  Figure 2 illustrates the current proportion of teachers in domestic colleges and universities who accept employment guidance training courses.

The employment guidance system of college students can fully play its role when a professional guidance team with the strong business ability and a sense of responsibility is established. The employment guidance work in colleges and universities should change the ideological concept of sitting still. They should provide services to students and comprehensively consider the employment mood of graduates and the talent needs of enterprises and institutions. They should provide opportunities for two sides to communicate, so the employment guidance of graduates can be carried out in an orderly manner. As the staff of the employment service system of colleges and universities, they should enhance their professional level from various aspects and provide effective recruitment information for graduates. In addition, they should continuously learn business knowledge and improve their enthusiasm for serving students. They should also improve their connection and communication skills with enterprises and other units. Besides, their ability to analyze, organize, and classify information should be improved.

It can be seen that only about 39% of teachers have received training, and only 13% of teachers have received employment training twice or more. This data shows that although the school attaches great importance to the construction of applied teachers, it has not invested enough in constructing employment guidance teachers. In particular, the opportunities for professional training and practical investigation of serving teachers are still limited in the actual teaching process of employment guidance courses, which is related to the school's investment in practice. Therefore, strengthening teachers' employment training courses is also a critical measure to improve the employment quality of college graduates.

Graduate students are the main body of employment. Sometimes, teachers have to undertake cumbersome teaching management tasks and pressure. Some instructors also serve as vocational counselors. They have to complete their tasks and spend extra time and energy preparing employment guidance courses. Considering comprehensively, it is more effective to improve the employability of graduates, the main body of employment, than improve the requirements for teachers.

### 2.2. Way of Integrating Deep Learning into College Students' Employment Training

Lv and Qiao (2020) pointed out that the essence of deep learning is a learning process with critical thinking on the new knowledge based on the understanding of ordinary learning. Applying it to the original identity structure makes it possible to connect thinking among many pieces of knowledge and transfer existing concepts to new scenarios. Here, a new theoretical concept of deep learning is proposed through analyzing and integrating the existing basic concepts of deep learning [13]. Deep learning refers to that with the help of teachers in class, students change from passive acceptance of knowledge to active exploration, understanding, and application of new knowledge and constantly reflect on new things and themselves in connection with their existing concepts. In this way, they can put forward their brand-new understanding and cognition to students and teachers and apply the knowledge learned in class to solve problems in real life. Deep learning can cultivate students to learn independently, cooperate with others, and use knowledge to solve problems rather than master the core theory of knowledge by rote learning. From the perspective of the required learning abilities, deep learning generally has the thinking characteristics summarized in Table 1.

At present, most employment guidance methods for college students use superficial learning methods. There is a big gap between superficial and deep learning in learning purpose, motivation, concentration, learning things, teaching methods, and final results [14], as shown in Table 2.

Unlike superficial learning, deep learning adopts different learning contents and teaching processes for different learning stages of students and helps learners transition from shallow and straightforward knowledge to deep and complicated knowledge. In this process, they are assisted by teachers [15]. In short, superficial learning is aimed at the learning foundation, while deep learning aims to deploy high-level deployment.  Figure 3 displays the special relationship between superficial learning and deep learning.

Deep learning can help students deeply understand and further expand basic knowledge and carry out active learning combined with actual deep situations and their conditions. Compared with superficial learning, it is more suitable to be used in college graduates' employment quality training strategy. Deep learning methods can reduce the burden on teachers and shift the protagonist of the teaching to the students themselves. After all, it is the graduates who need employment. Making students aware of the importance of employment quality and employment skills earlier can better help college graduates improve their abilities [16].

### 2.3. Employment Training Model of College Students Combined with Deep Learning

The school also focuses on cultivating students' various practical abilities in addition to specialized knowledge, including expression and communication ability, language communication ability, group cooperation ability, skill operation ability, and front-line management ability, highlighting the practicability of teaching [17]. Considering the unique object of employment guidance in higher vocational colleges, colleges and universities must pay attention to the preparation of college students before employment, that is, the guidance in the employment preparation period. Employment guidance aims to shape students' personality and survival ability, enable students to accept different teaching processes according to different expression characteristics of their learning stages and understand all kinds of professional abilities and personal quality requirements of their expected career, and trigger students to standardize their learning methods and learning ability and improve their self-quality. Therefore, the correct and effective teaching process and method can connect students with the professional needs of the society like a network and furnish students with opportunities to give full play of their talent [18].  Figure 4 reveals several training objectives of the employment training system suitable for college graduates.

The existing employment guidance course setting system should be optimized to strengthen the teaching effect of employment guidance courses. Sound system construction is a basis for the effective development of employment guidance work. Higher vocational colleges should combine policy theory education and practical guidance, cultivate students' employment awareness, and trigger students' learning motivation for job hunting to the greatest extent. Meanwhile, they shall assist students in planning their employment process, improve students' professional skills and application skills, and help students prepare for the fierce social competition [19]. The employment training system of college students shown in Figure 5 via deep learning combined with the school situation can play a significant role.

The teaching strategy structure must conform to the teaching objectives and tasks, take students as the center, and flexibly select and integrate teaching organization forms, teaching methods, and technologies to fundamentally regulate and control teaching to improve students' employment skills. To connect with famous international universities, the teaching of Chinese application-oriented universities should face the diversified talent needs of the whole society and establish an innovative concept and strategy of training all new applied talents. Domestic colleges and universities should provide the country with comprehensive talents with rich professional knowledge reserves, outstanding comprehensive practical ability, high individual quality, and problem-solving ability [20].

### 2.4. Design of the Employment Quality Evaluation Questionnaire for College Students

A questionnaire has a very high usage rate as a measure that can intuitively reflect the situation of the experimental object. The questionnaire designed here aims to verify the performance and applicability of the employment training model [21] and understand the guidance of teachers for students in the process of teaching and students' learning status and attitudes towards employment. This information can be used as the basis for research and analysis and can also be combined with relevant educational theoretical knowledge and teaching guiding ideology to put forward some new guiding strategies for students' in-depth learning and courses. Based on the three-point scale method, the questionnaire expresses the respondents' attitude towards the questions into five options according to different degrees: strongly disagree, disagree, neutral, slightly agree, and quite agree. Each option is assigned different points: strongly disagree = 1, disagree = 2, neutral = 3, slightly agree = 4, and quite agree = 5. The questionnaire is designed from four aspects: learning motivation, concentration, teaching process, and final results.  Table 3 shows the content of the questionnaire.

After the design, the questionnaire needs to be tested for validity and reliability. First, it is necessary to determine the number of survey objects, that is, to select the appropriate number of samples. Too many samples will waste resources, while too few samples will lead to inaccurate survey results. Therefore, oversampling or undersampling processing is required for the unbalanced data in the experiment [22]. Oversampling refers to the rearrangement of data arrangement rules to solve the unbalanced data, that is, to improve the classification performance of a small number of samples by adding a small number of samples. However, oversampling has the problem of overfitting due to the additional data that has not been accurately tested. The appropriate sample volume is calculated according to

(1) $$\begin{array}{c} n=\frac{1}{\left(1/N+d^{2}/\mu_{\alpha /2}^{2}\times s^{2}\right)}. \end{array}$$

(1) can be simplified as

(2) $$\begin{array}{c} n=\frac{N\mu_{\alpha /2}^{2}\times s^{2}}{Nd^{2}+\mu_{\alpha /2}^{2}\times s^{2}}. \end{array}$$

In equation (2), *n* is the sample volume. *d* is the limit sampling error under the allowable conditions, which is a constant determined according to the field conditions. *µ* is the particle size of the equivalent volume particle. *N* represents the overall scale of the survey objects, that is, the total number of all survey objects that can be selected as survey objects. In addition, the principle of this algorithm is to take samples from adjacent random samples and take a few points on the connecting line of two samples as newly synthesized samples. The essence of undersampling is to extract some samples from a large number of data samples as a representative. This method usually leads to the loss of some vital data information and cannot make full use of data information. Therefore, a clustering-based downsampling method is proposed here to solve this problem. In *s*^2^=*px*(1 − *p*), *p* is the proportion of the sample, which is generally 0.5. It is necessary to evaluate the surveyed model to obtain the prediction result. Comparing the predicted value with the actual value can judge the generalization ability of the model. The *a* coefficient is often used for the validity test, as shown in thefollowing equation:

(3) $$\begin{array}{c} \alpha =\left[\frac{N}{N-1}\right]\left(\frac{1-\sum Si^{2}}{S^{2}}\right). \end{array}$$

In (3), *N* denotes the total number of survey questions in the questionnaire, ∑*Si*^2^ represents the variance sum of all questions, and *S*^2^ stands for the total score variance of all questions. Reliability is the degree of reliability of a test. It mainly shows the continuity, consistency, reproduction, and stability of test results. It also indicates whether the test results reflect the stable and consistent true characteristics of the subjects. The same thing is measured over and over again, and the result should always remain the same. The most commonly used measure is the Cronbach coefficient. In general, the internal reliability of the scale is mainly considered—whether there is a high internal consistency between items. It is generally believed that the reliability coefficient should be between 0 and 1. If the reliability coefficient of the scale is above 0.9, the reliability of the scale is very good. If the reliability coefficient of the scale is between 0.8 and 0.9, the reliability of the scale is acceptable.

## 3. Results

### 3.1. Validity Test Results of the Questionnaire

Generally, when the *a* coefficient is larger than 0.9, the question and scoring design of the questionnaire is rational, and the survey is practicable. After calculation, the *a* coefficient is 0.928 > 0.9, indicating that the questionnaire validity is excellent. Then, teachers and professors in a university are invited to judge the practicality of the questionnaire questions.  Table 4 shows the evaluation results.

The results in Table 4 indicate that the questions are well set up and can be used as the basis for investigations. Subsequently, 80 questionnaires are distributed randomly to students of four grades in colleges and universities in a specific place. A total of 76 covers are collected, including 73 valid questionnaires. The data processing software SPSS25 is used to process the results of the questionnaires counted as the experimental results.

### 3.2. Learning Results of Male and Female Students Based on the Employment Quality Evaluation Model

As Figure 6 presents, in this survey, the employment quality guidance model is judged and counted according to different genders. The statistics are organized in four directions: learning motivation, attention, teaching process, and final result. Among the 73 valid questionnaires, there were 12 male students, accounting for about 16%, and 61 female students, accounting for about 84%.

In Figure 7, the Measure of Effectiveness (MOE) values of the two significantly related dimensions of learning things and evaluation strategies are 0.0521 and 0.0492, respectively, both less than 0.06. The results indicate that gender is slightly correlated to teaching content and evaluation methods. In the evaluation of male students, the average values of learning motivation, concentration, teaching process, and final result are 3.3576, 3.1473, 3.4351, and 3.4865, respectively; the standard deviation values are 0.7354, 0.8246, 0.7545, and 0.5584. The mean MOE of female students is 3.8464, 3.1557, 3.4257, and 3.4566, and the standard deviation is 0.6188, 0.6483, 0.5844, and 0.4384. For employment guidance and subsequent employment quality, male and female students are very similar in terms of employment quality from the above data. This means that the employment guidance and employment quality are closely related to the school's employment curriculum. Therefore, schools need to further develop career guidance courses. The results suggest that gender differences do not affect the employment guidance model and the final employment quality. It can also prove that when male and female students conduct deep learning, there will not be a big difference in results due to personal habits.

### 3.3. Numerical Analysis of Each Dimension

This section is the regression analysis to determine the degree of influence of multiple variables on a single variable to prove the significant relationship between the independent and dependent variables. Therefore, according to the calculation and analysis results, the learning result is the dependent variable, and the learning motivation, concentration, and the teaching process are used as independent variables. The results are shown in Figures 8.

According to the data in Figures 8 and 9, the *P* values of learning motivation, concentration, and teaching process are all less than 0.01, indicating that the three perspectives have a certain degree of influence on the learning results. In addition, the nonstandard coefficients in Figure 8 are 0.0633, 0.1834, and 10.3491, respectively. The standard deviations in Figure 9 are 0.0181, 0.0174, and 0.0223. This reveals that its condition is good, and its standard coefficients are 0.0912, 0.2836, and 0.4897, which are similar to the data in Figure 8. Besides, the Unstandardized Coefficients B of the three dimensions are all greater than 0, proving that the three dimensions positively impact the learning results. In other words, the more sufficient the learning motivation, the more profound the degree of concentration, the better the teaching process, and the better the learning results. In addition, the numerable value of the learning results is equal to 0.0633 (learning motivation) plus 0.1834 (concentration) plus 0.3491 (teaching process), and the standard deviation in Figure 9 is similar to the data in Figure 8. It can be judged that the teaching process has the hugest impact on the learning results. Therefore, taking measures suitable for students during the teaching process is conducive to learning concentration and motivation, worthy of innovative research.

## 4. Conclusion

The following are some guiding suggestions for the employment of graduates through the analysis of the results of the questionnaire:

The competition mechanism has penetrated all areas of society and the entire process of life. Students begin to compete for academic performance from entering the campus. Everyone wants to get good grades. At the university level, the competition is intense. Evaluation of three-good students and outstanding graduates and graduate recommendations are related to the competition. However, college students' sense of competition has not been strengthened. Some college students seem helpless in competition. Today's deepening of reforms puts forward urgent requirements for college students to strengthen their sense of competition and also provides an objective environment. Meeting new challenges and strengthening the sense of competition are the most basic psychological preparations for college students before choosing a career.

Guidance on employability skills for graduates should be provided in time. This paper employs deep learning technology as an instructional technology and integrates it into college students' job-seeking education. Firstly, the social status quo of graduates' employment difficulties is expounded from the research structure of the paper. The various definitions of literacy and core literacy are all applied to new situations or future development. Transfer refers to the knowledge gained by completing a task in one context and the ability to apply it to another context and another task. The concept of core literacy originates from the challenges of adapting to the constantly updated and changing information age and knowledge society. It refers to an individual's ability to solve complex problems in unpredictable. Therefore, most core competency frameworks include transferable competencies, such as creative and critical thinking, problem-solving, and new product development. Besides, a questionnaire on college students' employment quality and deep learning effect is designed from four perspectives based on the influencing factors of deep learning on learning results: learning motivation, concentration, teaching process, and final results. In the experimental link, the two groups of male and female students are compared through various data analyses and processing. It is found that gender does not have a significant impact on the effect of deep learning and employment quality due to different learning methods. The computable value of learning outcomes is equal to 0.0633 (learning motivation) plus 0.1834 (attention) plus 0.3491 (teaching process). The standard deviation in Figure 9 is similar to the data in Figure 8. In conclusion, the teaching process has the greatest impact on learning outcomes. In the subsequent multifactor influence research, it is found that the teaching process has the most significant impact on the employment quality and the effect of deep learning among the learning motivation, attention, and teaching process. Therefore, schools need to fundamentally improve students' in-depth learning effect and employment quality starting with professional employment teaching guidance. Corresponding teaching strategies are proposed for students of specific majors to improve students' learning motivation and strengthen their learning focus. The shortcoming of this paper is the small number of questionnaires and valuable experimental samples. It affects the accuracy of the response rate, thereby affecting the sample size. In the process of calculating samples, the following important aspects should also be considered. First, sampling inference must be done to ensure the accuracy of the sampling rate. Second, the overall degree of variation is determined according to the size of the variance. Third, the amount of sampling depends on the size of the variance. If the variance is large, take more samples. If the variance is small, take fewer samples. Fourth, the number of samples is also related to the funding situation, including the expenses of investigators, the expenses of investigation channels, and the cost of questionnaires. The sample size depends on the estimated domain. In short, the determination of sample size should follow the principle of interaction between precision and cost. The cost is certain, and the accuracy is the highest. The accuracy is certain, and the cost is the lowest. Therefore, the follow-up research will expand the scale of research objects to make the research results more in line with the current situation.

## Figures and Tables

**Figure 1:** The vicious circle of employment.

**Figure 2:** Teachers' acceptance of employment guidance training courses.

**Figure 3:** Relationship between superficial learning and deep learning.

**Figure 4:** Employment training goals for college graduates.

**Figure 5:** Employment training system based on school scenarios combined with deep learning.

**Figure 6:** Evaluation results of male and female students on the employment guidance model. (a) The data result of male students. (b) The data result of female students.

**Figure 7:** The measure of effectiveness of the judge strategy and learning things.

**Figure 8:** Multidimensional influence degree analysis.

**Figure 9:** Multidimensional standard error analysis.

**Table 1:** Thinking characteristics of deep learning.

Concept	Content
Student-centered	Learners are responsible for themselves and should engage in learning with interest in improving the quality and effect of learning. Teachers guide students with the main purpose of meeting their needs.
Life-long learning	Shallow learning only pays attention to the immediate task and lacks reflection on learning and evaluation of results. On the contrary, deep learning requires timely summarization and criticism of mistakes in learning and continuous improvement to proficiency.
Comprehension capability	Shallow learning is passive learning. However, deep learning focuses on understanding and treating problems and problems with a skeptical attitude, which can increase one's objective evaluation and achieve the purpose of deep thinking.
Integration capability	Deep learning emphasizes integrating new knowledge and old knowledge, which requires a broader acquisition of knowledge and establishing its knowledge base.
Conversion capability	Students need to strengthen self-consciousness, improve the ability of self-understanding, self-examination, self-evaluation, self-control, and transformation, and reflect and summarize the knowledge results established.
Application ability	Superficial learning methods only focus on ending the immediate problems with mechanical methods. Deep learning cultivates students' ability to use their own knowledge comprehensively.
Problem-solving ability	Superficial learning can only solve written problems with scattered knowledge. In contrast, deep learning emphasizes applying the knowledge learned in real life to solve complex problems in practical situations.
High-latitude thinking	Current superficial learning methods still emphasize low-level goals, such as memorizing written knowledge and understanding surface meaning. Deep learning focuses on combining and applying knowledge with real life and creating things of higher value, focusing on knowledge application and high-latitude ideas of improving learning effectiveness.

**Table 2:** Gaps between superficial learning and deep learning.

Feature	Superficial learning	Deep learning
Learning purpose	To complete the basic tasks assigned by the teacher	Focusing on advanced development of basic knowledge
Learning motivation	Passive learning at the request of family and teachers	Spontaneous learning triggered by students' interests
Concentration	Students are passive and have a low concentration.	Students are in an active learning state
Learn content	Boring written knowledge	Knowledge combining questions with real-world situations
Teaching methods	The current common teaching strategy of one teacher and many students	Students are the main body; teachers are the assistants, which focuses on ability development
Final results	Student achievement is uneven, and the gap is too large	Students can use concepts flexibly to solve practical difficulties

**Table 3:** Questionnaire content.

Basic information						
Gender		A. Male		B. female		

Grade		A. Freshman	B. Sophomore	C. Junior	D. Senior	

Major						

Class ranking		A. Top 5%	B. 5%–30%	C. 30%–60%	D. 60%–90%	E. The last 10%

Question number	Question content	Strongly disagree	Not agree	Neutral	Slightly agreeable	Quite agree

Learning motivation						
1	I study hard just to get a job.	A	B	C	D	E
2	I think it makes sense to adopt deep learning.	A	B	C	D	E
Concentration						
3	I will do a preview before class.	A	B	C	D	E
4	My purpose is clear when I study.	A	B	C	D	E
5	I will actively answer the teacher's questions.	A	B	C	D	E
Teaching process						
6	I can use the teacher's method.	A	B	C	D	E
7	I can seek answers through the internet.	A	B	C	D	E
8	I will ask my teachers and classmates for questions.	A	B	C	D	E
Final results						
9	I think this way of learning is significantly beneficial to my employment.	A	B	C	D	E
10	I am able to apply the new knowledge in the classroom flexibly in my life.	A	B	C	D	E
11	I can get the satisfaction of serious study.	A	B	C	D	E

**Table 4:** Questionnaire evaluation results.

Judge	Evaluation criteria		
	Very perfect (%)	Relatively perfect (%)	Imperfect (%)
Teacher A	69	21	10
Teacher B	34	60	6
Professor A	50	46	4
Professor B	85	3	12

## Data Availability

The data used to support the findings of this study are included within the article.
